This article has been retracted.

# Development of Machine Learning-Based Ideas for Teaching Physical Education and Health

**DOI:** 10.1155/2022/4418606

**Published:** 2022-08-17

**Authors:** Weiyu Yin, Sheng Li, Cuiyi Han

**Affiliations:** ^1^Graduate School, Shandong Sport University, Jinan, 250102 Shandong, China; ^2^School of Wushu, Shandong Sport University, Jinan, 250102 Shandong, China

## Abstract

With various social pressures and the lack of knowledge about physical health, students have poor physical education quality and insufficient knowledge acquisition about physical health. Traditional physical health teaching is a process in which the teacher tells the theory of physical health and students passively accept it, which leads to physical health problems such as low learning efficiency of students' physical health knowledge and low interest in learning physical health knowledge. With the emphasis on physical health teaching and the development of technologies such as machine learning, machine learning is used to analyze the problems of physical health teaching and help students to learn physical health better to improve the efficiency of physical health teaching. The results of this paper show that the machine learning-based physical education and traditional physical education can reduce the injury rate of students' sports by 7.7% compared with traditional physical education, make students' interest in physical education and health learning reach 53.3%, and improve the efficiency of physical education and health learning. There is a degree of students' acquisition of physical health knowledge. The change from traditional physical health teaching ideology to machine learning-based physical education ideology can improve the teaching efficiency of physical health teaching, allow students to acquire more physical health knowledge, and effectively reduce the risk of students' injuries in sports.

## 1. Introduction

With the development of machine learning and other technologies, it has a significant impact on the production and life of society as well as education. People's thinking about physical health education has also changed. The traditional idea of physical health education belongs to the classroom lecture mode, in which physical education teachers instill physical education knowledge to students and teach little about health concepts. Students are in the process of receiving physical education knowledge passively for a long time, which leads to the lack of active learning ability for physical health knowledge, and the defects of traditional physical health education such as single content and high repetitiveness make some students averse to physical health. Traditional physical health education ideology makes students' physical health knowledge acquisition insufficient, average body quality decreases, and physical health teaching efficiency decreases. Therefore, it is crucial to change the idea of physical health education. Machine learning has a good ability of classification and prediction as well as data analysis, and machine learning technology is used to analyze the substandard physical action of students, predict students' physical hobby, and motivate students to learn physical health. The education of students' physical health requires a fundamental change in the thinking of physical health education, and the use of machine learning technology makes the teaching of physical health more efficient. Therefore, this paper has research significance.

Due to the lack of students' physical health knowledge, some researchers have improved students' lack of physical health knowledge through physical health instruction. Among them, Hodges t al. showed that the majority of students lack physical health knowledge, and that enhancing physical health instruction can improve students' physical health knowledge [1]. Dunleavy et al. pointed out that physical health instruction can promote students' motivation and initiative towards physical health [2]. Thompson et al., who conducted a study in collaboration with experts in psychological aspects, stated that physical health instruction can not only reduce students' chances of sports injuries but also enhance students' mental health [3]. Chun and Yin found that students' physical health is poor, and physical health education is important for improving students' physical fitness [4]. The Bartram et al. experiment compared those who received physical health instruction with those who did not and found that those who received physical health instruction have better physical fitness [5]. Although the physical health teaching approach can improve the efficiency of physical health teaching to a certain extent and help students acquire physical health knowledge, there is a lack of intelligent technology to assist physical health teaching [6].

Machine learning can be a good way to analyze and predict physical health teaching data and use machine learning to assist in analyzing physical health teaching [7]. Among them, Li used machine learning that can analyze various problems in physical health teaching and greatly improve the quality of physical health teaching and the efficiency of students' learning [8]. Zhang showed that the machine learning-based approach to physical health teaching can effectively develop students' knowledge in physical health [9]. Hou stated that using techniques such as machine learning technology to analyze students' physical health education can develop appropriate physical health teaching plans to help students better acquire knowledge about physical health [10]. Zhang and Min stated that traditional physical health teaching methods cannot meet the development of physical health curriculum, and that the combination of technologies such as machine learning and physical health teaching is the trend of physical health development [11]. Yang stated that physical health teaching using machine learning can improve students' physical fitness [12]. Although the use of technologies such as machine learning to assist in teaching physical health can be effective in improving students' physical fitness and help them learn physical health more effectively, the use of machine learning to analyze predictions is not optimal [13].

This paper uses machine learning techniques to analyze physical health teaching problems and predict the learning status of students conducting physical education, so as to develop personalized physical health teaching programs and improve the efficiency of students conducting physical health learning. The innovation points of this paper are as follows: (1) to assist physical health teaching by machine learning and (2) comparing machine learning-based physical education and health teaching with traditional physical education and health teaching to highlight the advantages of machine learning-based physical education and health teaching.

## 2. Machine Learning-Based Approach to Teaching Physical Health

Machine learning-based physical health teaching is used to improve the efficiency of physical health teaching by analyzing students' learning status of physical health learning and students' feedback on physical health teaching to change the way of physical health teaching and improve students' physical training ability. The model of physical health teaching based on machine learning is shown in Figure 1.

Machine learning predicts the output of the system by training the samples. Its principle is to find the dependence between the independent variable *U* and the dependent variable *V*, that is, to find the probability of *f*(*U*, *V*). That is, according to *n* samples (*u*_1_, *v*_1_), (*u*_2_, *v*_2_), ⋯, (*u*_*n*_, *v*_*n*_), a function {*f*(*u*, *w*)} is selected to find the optimal solution *f*(*u*, *w*_0_), and the risk value *K*(*w*) is the lowest.

(1) $$\begin{array}{c} K\left(w\right)=\int D\left(v,f\left(u,w\right)\right)dF\left(u,v\right). \end{array}$$

In equation (1), *f*(*u*, *w*) denotes the prediction function, *w* is the parameter to be determined, and *D*(*v*, *f*(*u*, *w*)) is the loss of the prediction made by *f*(*u*, *w*) for *v*.

The core of machine learning is to train the observed data and predict to get the accurate data, and there are many methods to construct the prediction model for machine learning, among which, BP neural network, support vector machine, and plain Bayes are good regression prediction models [14, 15].

### 2.1. BP Neural Network Method

BP neural network is a type of artificial neural network, which is an intelligent model designed to simulate the processing computation of the human brain [16]. With a processing structure similar to that of the human brain, BP neural networks have superb learning and computational capabilities and have the ability to predict and analyze students' learning status.

#### 2.1.1. Neurons

Neurons are the most basic component unit of BP neural network and the basis of information processing. The information processing of BP neural network goes through neurons, and the weighted average of the outputs of all neurons is the output of BP neural network. The structure of neurons is shown in Figure 2.

As can be seen from Figure 2, the neuron needs to process many input signals. Let the input signal of the neuron be (*x*_1_, *x*_2_, ⋯, *x*_*n*_) and the connection weights between the neuron and the input signal be *W* = (*w*_1_, *w*_2_, ⋯, *w*_*n*_), and the signal processing process of the neuron is to sum the product of the input signal and the connection weights. The result of the neuron after processing is

(2) $$\begin{array}{c} s=\overset{n}{\underset{i=1}{\sum }}w_{i}x_{i}. \end{array}$$

The result of the neuron processing is then passed into the *f* function and finally output. *f* function is the activation function.

(3) $$\begin{array}{c} f\left(s\right)=\frac{1}{1+e^{-s}}. \end{array}$$

#### 2.1.2. BP Neural Network Structure

Different structures of neurons lead to different structures of neural networks. BP neural network is a multilayer feedforward network, which has the advantages of simple network structure, strong learning ability, and wide application range. It is very suitable for dealing with complex data structures and analyzing and predicting nonlinear problems, a good analysis of sports health teaching [17].

BP neural network is a three-layer structure model, where the information arrives first as the input layer, the information output as the output layer, and the middle structure as the hidden layer. The structure of BP neural network is shown in Figure 3.

As can be seen in Figure 3, let the input signal be *X* = (*x*_1_, *x*_2_,⋯,*x*_*n*_)^*T*^, the output of the implicit layer be *Y* = (*y*_1_, *y*_2_,⋯,*y*_*m*_)^*T*^, the output of the output layer be represented as *U* = (*u*_1_, *u*_2_,⋯,*u*_*k*_)^*T*^, the connection weight of the input layer to the implicit layer be *V* = (*v*_1_, *v*_2_,⋯,*v*_*m*_)^*T*^, and the connection weight of the implicit layer to the output layer be*W* = (*w*_1_, *w*_2_,⋯,*w*_*k*_)^*T*^.

The output layer is expressed as

(4) $$\begin{array}{c} U_{t}=f\left({\text{net}}_{t}\right). \end{array}$$

In equation (4), the range of values of *t* is (1, 2, ⋯, *k*)_,_ and net_t_ represents the processing of the *t*-th neuron in the output layer.

(5) $$\begin{array}{c} {\text{net}}_{t}=\overset{m}{\underset{j=0}{\sum }}w_{t}y_{j}. \end{array}$$

The implicit layer is expressed as

(6) $$\begin{array}{c} y_{j}=f\left({\text{net}}_{j}\right). \end{array}$$

In equation (6), *j* takes values in the range (1, 2, ⋯, *m*)_,_ and net*_j_* represents the processing of the *j*-th neuron in the hidden layer.

(7) $$\begin{array}{c} {\text{net}}_{j}=\overset{m}{\underset{i=0}{\sum }}v_{ij}x_{i}. \end{array}$$

#### 2.1.3. The Learning Process of BP Neural Network

The learning process of BP neural network is also the process of approaching the actual output of BP neural network to the desired output, which is composed of forward propagation of information and backward transmission of error [18]. The backward transmission of error is the process by which the error of the output layer goes through the hidden layer and then to the input layer, and the structure of the neural network is adjusted by adjusting the threshold of the neurons in each layer. Thus, the output of the neural network is changed and finally, the error is brought to an acceptable range.

The reverse transmission of errors modulates neurons as follows.

Let *U*_*i*_ be the output of the *i*-th neuron, *R*_*j*_ be the input of the *j*-th neuron, and *v*_*ij*_ be the connection weight between the *i*-th and *j*-th neurons. The *j*-th neuron has the following relationship.

(8) $$\begin{array}{c} R_{j}=\underset{i}{\sum }v_{ij}U_{i}. \end{array}$$

Then, the error of the BP neural network is expressed as

(9) $$\begin{array}{c} E=\frac{1}{2}\underset{k}{\sum }{\left(y_{k}^{q}-y_{k}^{s}\right)}^{2}. \end{array}$$

In equation (9), *y*_*k*_^*q*^ denotes the desired output of the *k*-th neuron, *y*_*k*_^*s*^ denotes the actual output of the *k*-th neuron, and *E* represents the error of the BP neural network.

Let the connection weights from the *j*-th neuron to the *k*-th neuron at moments *t* and *t* + 1 be *v*_*jk*_(*t*) and *v*_*jk*_(*t* + 1), respectively, and then there is the following relationship.

(10) $$\begin{array}{c} v_{jk}\left(t+1\right)=v_{jk}\left(t\right)+\Delta v_{jk}. \end{array}$$

In equation (10), Δ*v*_*jk*_ denotes the connection weight of the *j*-th neuron to the *k*-th neuron for this variable.

The core of BP neural network learning is the back propagation of error. The network structure is adjusted by changing the connection weights between neurons. Therefore, finding Δ*v*_*jk*_ is the key to the learning of BP neural network. The gradient descent method is used to solve the minimum error of *E* and Δ*v*_*jk*_.

(11) $$\begin{array}{c} \Delta v_{jk}=-z\frac{\partial E}{\partial v_{jk}}. \end{array}$$

In equation (11), *z* denotes the error factor.

Organizing equations (11) and (8) yields as follows:

(12) $$\begin{array}{c} \Delta v_{jk}=-z\frac{\partial E}{\partial R_{k}}\frac{\partial R_{k}}{\partial v_{jk}}. \end{array}$$

Solve *∂E*/*∂R*_*k*_ and *∂R*_*k*_/*∂v*_*jk*_:

(13) $$\begin{array}{c} \frac{\partial R_{k}}{\partial v_{jk}}=U_{j}, \end{array}$$

(14) $$\begin{array}{c} \frac{\partial E}{\partial R_{k}}=-\left(y_{k}^{q}-y_{k}^{s}\right)f^{\prime }\left(R_{k}\right). \end{array}$$

BP neural networks have powerful regression analysis capabilities and can predict quite accurate results after only a certain amount of data training [19].

### 2.2. Support Vector Machine Method

Statistical learning methods are a way in which a system can make accurate predictive estimates with a limited number of training samples [20]. Support vector machine is a method in statistical learning that regulates the optimal relationship between learning ability and learning accuracy based on a limited number of samples. The principle of support vector machines is to create a classification hyperplane that categorize physical health teaching problems into certain categories.

The support vector machine is based on statistical learning methods to find the optimal classification surface to minimize the error of the sample data from the found classification surface, and the classification model of the support vector machine is shown in Figure 4.

The classification prediction principle of the support vector machine is based on a finite set of training samples with *m* training samples {(*u*_1_, *v*_1_), (*u*_2_, *v*_2_), ⋯, (*u*_*m*_, *v*_*m*_)}, where *u*_*i*_ is the *i*-th input data, and *v*_*i*_ is the *i*-th output data [21].

The support vector machine linear regression function is

(15) $$\begin{array}{c} f\left(x\right)=a\phi \left(x\right)+b. \end{array}$$

In equation (15), *ϕ*(*x*) is the mapping function.

Let *r* be the error spacing, and then the linear insensitivity function is expressed as

(16) $$\begin{array}{c} G\left(f\left(x\right),y,r\right)=\left\{\begin{array}{c} \left|y-f\left(x\right)\right|-r,\left|y-f\left(x\right)\right|>r\\ 0,\text{other} \end{array}\right.. \end{array}$$

In equation (16), *y* is the corresponding output value of the input data *x*.

Let the slack variables be *h*_*i*_ and *h*_*i*_′, and then finding the values of the regression parameters *a* and *b* can be converted to

(17) $$\begin{array}{c} \left\{\min\frac{1}{2}{\left\|a\right\|}^{2}+Q\overset{m}{\underset{i=1}{\sum }}\left(h_{i}+h_{i}^{\prime }\right)\left\{\begin{array}{c} y_{i}-a\phi \left(x_{i}\right)-b\leq r+h_{i},i=1,2,\cdots ,m,\\ -y_{i}+a\phi \left(x_{i}\right)+b\leq r+h_{i}^{\prime },\\ h_{i},h_{i}^{\prime }\geq 0. \end{array}\right.\right. \end{array}$$

In equation (17), *Q* denotes the penalty factor, and a larger *Q* indicates a larger penalty for samples with larger error than r.

Let the kernel function be *D*(*x*), and then the regression function is expressed as

(18) $$\begin{array}{c} f\left(x\right)=\overset{m}{\underset{i=1}{\sum }}a^{\prime }D\left(x\right)+b^{\prime }. \end{array}$$

In equation (18), *a*′ and *b*′ are the solutions of the regression parameters, respectively.

### 2.3. Plain Bayesian Approach

The plain Bayesian classification algorithm is based on the features of the data, has the advantages of high classification accuracy and fast computation, and is a common classification algorithm used in machine learning, and it can accurately classify the problems of sports health teaching [22].

#### 2.3.1. Bayes' Theorem

Let the sample set of the experiment be *K*, *C* be the experimental event, and *D*_1_, *D*_2_, ⋯, *D*_*n*_ be the event set of *K*, and each event in the event set has a probability other than zero. Then,

(19) $$\begin{array}{c} P\left(C\right)=P\left(C\left|D_{1}\right.\right)P\left(D_{1}\right)+P\left(C\left|D_{2}\right.\right)P\left(D_{2}\right)+\cdots +P\left(C\left|D_{n}\right.\right)P\left(D_{n}\right)=\overset{n}{\underset{i=1}{\sum }}P\left(C\left|D_{i}\right.\right)P\left(D_{i}\right). \end{array}$$

The formulation process of equation (19) is the full probability formula.

(20) $$\begin{array}{c} P\left(D_{i}\left|C\right.\right)=\frac{P\left(C\left|D_{i}\right.\right)P\left(D_{i}\right)}{\sum_{j}^{n}P\left(C\left|D_{j}\right.\right)P\left(D_{j}\right)}. \end{array}$$

In equation (20), *i*, *j* ∈ (1, 2, ⋯, *n*).

#### 2.3.2. Plain Bayesian Classification Model

Plain Bayesian classification is usually performed using a plain Bayesian parser, in which the input set is made to be {*B*_1_, *B*_2_, ⋯, *B*_*n*_, *C*}, and the plain Bayesian classifier model is shown in Figure 5.

Let the input data sample set be *S* = {*s*_1_, *s*_2_, ⋯, *s*_*n*_} and the posterior probability be*P*(*B*_*i*_|*S*).

A parsimonious analysis of conditionally independent data has been presented, viz.,

(21) $$\begin{array}{c} P\left(S\left|B_{i}\right.\right)=\overset{n}{\underset{k=1}{\prod }}P\left(s_{k}\left|B_{i}\right.\right). \end{array}$$

#### 2.3.3. Bayesian Classification Model with Expanded Tree Shape

The independence between conditions of the plain Bayesian is strong, and since the subnodes of the plain Bayesian are covered by attribute nodes, enhancing the correlation between subnodes can reduce the independence between conditions [23]. The Bayesian classification model with an expanded tree shape is shown in Figure 6.

Let the child node be {*B*_1_, *B*_2_, ⋯, *B*_*n*_}, the attribute node be *C*, and the input data sample set be*S* = {*s*_1_, *s*_2_, ⋯, *s*_*n*_}.

Then, the function of child nodes passing information to each other is

(22) $$\begin{array}{c} H_{p}\left(B_{i},B_{j}\left|Z\right.\right)=\underset{s,y,z}{\sum }P\left(s_{i},s_{j},z\right)\log\frac{P\left(s_{i},s_{j}\left|z\right.\right)}{P\left(s_{i}\left|z\right.\right)P\left(s_{j}\left|z\right.\right)}. \end{array}$$

## 3. Experimental Data Comparing Machine Learning-Based Physical Education and Health Teaching with Traditional Physical Education and Health Teaching

### 3.1. Sample Data

In order to be able to better analyze the impact of machine learning-based teaching methods on physical health teaching, this paper compares physical health teaching based on machine learning with traditional physical health teaching, mainly through the form of comparative evaluation indicators [24]. Therefore, the selection of the experimental sample is especially critical to the comparison experiment, and the improper sample selection can easily lead to invalid comparison experiment. In order to make the sample sufficiently convincing, the sample should be randomly selected and randomly distributed over the whole segment of the sample.

Since the high school level is the stage that best reflects the quality of physical health instruction, an experiment will be conducted on high school physical health instruction. Twenty high schools will be selected for the experimental data, 10 of which will use machine learning-based physical health instruction while the other 10 high schools will use traditional physical health instruction. A questionnaire will be administered to 100 students in each of the three categories of senior high school, sophomore high school, and senior high school for a period of 3 months to investigate the indicators that reflect the quality of physical health teaching, and the results of the study are shown in Table 1.

The data in Table 1 shows that the six indicators studied to evaluate the quality of physical education, and health teaching had an average impact of 73.7%, 67%, and 73.3% on the three populations of seniors, juniors, and seniors, respectively.

### 3.2. Correlation Analysis of the Sample

When selecting indicators for evaluating the quality of physical health teaching, a correlation analysis of the sample of evaluation indicators and physical health teaching is required. Correlation analysis of the sample is used to determine the degree of correlation between the indicators and physical health instruction, and correlation analysis of the sample allows amplification of the main features of the physical health instruction experiment and makes it more useful to observe which indicators have an impact on physical health instruction [25]. The results of the correlation analysis of the evaluation indicators are shown in Table 2.

From the data in Table 2, it can be obtained that the highest correlation of students' physical education injury rate to physical health instruction was 0.264, and the lowest correlation was students' love for physical education [26]. The correlation degree of the first four evaluation indicators in Table 2 exceeded 0.2, while the correlation degree of the last two evaluation indicators were 0.026 and 0.034, respectively. Therefore, the last two evaluation indicators will not be used as indicators for evaluating physical health teaching.

### 3.3. Analysis of the Validity of the Sample

In order to test whether the first four indicators in Table 2 can compare two types of physical health instruction, the experiment will perform *k*-weight crossvalidation of the evaluation indicators and physical health instruction. Since the sample data for this experiment is not very large, the experiment uses a 5-fold crossvalidation method, which means that 240 of the data are the test set and the remaining 60 data are the test set, and the results of the experiment are the average of five experiments [27]. The results of the sample validity analysis are shown in Table 3.

From the data in Table 3, the highest validity in the machine learning-based physical health instruction was 88.4% for the acquisition of physical health knowledge, and the highest validity in the traditional physical health instruction was 86.2% for the students' interest in physical health learning. The average validity of the four evaluation indicators for the two types of physical health instruction was 82.4% and 80.0%, respectively. Since the average validity of both physical health instruction exceeded 80%, a comparative analysis of these four evaluation indicators could be conducted for both physical health instruction.

## 4. Physical Health Teaching Results and Discussion

Machine learning-based physical health teaching is based on techniques such as BP neural networks to analyze the state of students when they perform physical health teaching in order to predict and analyze to determine the most suitable physical health teaching method for students, while traditional physical health teaching uses the teacher-to-student indoctrination teaching method [28]. The experiment will compare the two physical health teaching methods in four aspects: students' physical injuries, students' level of interest in physical health learning, the efficiency of physical health teaching, and the degree of physical health knowledge acquisition.

### 4.1. Students' Sports Injuries

Students' physical education injury rate is a reflection of students' knowledge of physical education and health, and a low rate of students' physical education injury reflects good physical education and health teaching ability, while a high rate of students' physical education injury reflects poor physical education and health teaching ability. A 6-month experiment was conducted with 100 students in each of the three years of senior high school, sophomore high school, and junior high school, and the students' physical education injury rates were investigated at one-month intervals. The results of the comparison of the students' physical education injury rates between the two physical health teaching styles are shown in Figure 7.

From the analysis of the data in Figure 7, it can be seen that the PE injury rate of students in the machine learning-based PE health teaching model is gradually decreasing, while the PE injury rate of students in the traditional PE health teaching model is decreasing slowly and sometimes tends to increase. In the six-month experiment, the lowest average PE injury rate for students in the machine-learning-based physical health instruction group was 21% for seniors, while the average PE injury rate for seniors in the traditional physical health instruction was 30.2%, and machine learning-based physical health teaching has lower injury rates for students.

### 4.2. The Level of Students' Interest in Physical Health Learning

A good way of teaching physical health is to stimulate students' interest in physical health learning. Since the degree of interest of male and female students in physical health is not the same, the experiment was conducted separately for male and female students. The experimental time was set to 6 months to observe the students' interest in physical health learning under the two physical health teaching modes, and the experimental results of students' interest in physical health learning are shown in Figure 8.

From the analysis of the data in Figure 8, it can be seen that the level of interest of boys in physical health learning is generally a little more than that of girls, but both the level of interest in physical health learning and the growth degree of interest in physical health learning are better in the machine learning-based physical health teaching model than the traditional physical health teaching model, and the average interest of students in the two teaching models in physical health learning is 53.3% and 40.3%.

### 4.3. Efficiency of Physical Education and Health Teaching

The teaching efficiency of traditional physical health education is not very good because it is conducted in the form of teachers teaching students what to do. In order to effectively compare the differences in teaching efficiency between the two physical education modes, the experiment was carried out on three types of students in senior high school, sophomore high school, and senior high school, the teaching efficiency of the two kinds of physical health teaching was compared in one semester, the efficiency of physical health teaching was counted every 4 weeks interval, and the teaching efficiency of the two kinds of physical health teaching is shown in Figure 9.

From the analysis of the data in Figure 9, it can be obtained that the two physical health teaching methods have roughly similar trends among the three groups of students, but overall, the teaching efficiency of the machine learning-based physical health teaching is higher than the traditional physical health teaching, and the teaching efficiency of the senior students of the two physical health teaching methods is the highest, respectively: 66.5% and 49.3%.

### 4.4. Degree of Access to Physical Health Knowledge

Teaching physical health will improve students' acquisition of physical health knowledge, and the degree of acquisition of physical health knowledge is also a measure of how well a physical health teaching approach works. The experiment was conducted for three grades, senior high school, sophomore high school, and junior high school, and the students' acquisition of physical health knowledge was counted once a month for six months. The results of the degree of students' acquisition of physical health knowledge under the two types of physical health teaching are shown in Figure 10.

From the analysis of the data in Figure 10, it can be seen that the difference in the students' acquisition of physical health knowledge in the first two months under the two types of physical health instruction was not significant, but the growth rate of students' acquisition of physical health knowledge under the machine learning-based physical health instruction was much larger than that under the traditional model. The average degree of students' acquisition of physical health knowledge under the two types of physical health instruction was 73.2% and 63.9%, respectively, higher acquisition of sports knowledge based on machine learning.

### 4.5. Experimental Analysis

Through a comparative analysis of all aspects of the two physical health teaching methods, the experimental results show that the machine learning-based physical health teaching is better than the traditional physical health teaching mode in four aspects: students' physical injuries, students' degree of interest in physical health learning, the efficiency of physical health teaching, and students' acquisition of physical health knowledge, and the average comparison of the specific two methods of physical health teaching was as follows. The data are shown in Table 4.

## 5. Conclusions

By comparing four aspects of machine learning-based physical health instruction with traditional physical health instruction, the following conclusions were drawn: (1) students' interest level in physical health learning under the machine learning-based physical health instruction model was 53.3%, compared with 40.3% under traditional physical health instruction. The machine learning-based physical health teaching model can effectively reduce the probability of injury in students' sports, and the probability of injury in students' sports is reduced by 7.7% compared with the traditional physical health teaching. (2) Machine learning-based physical health teaching is 16.1% and 9.3% more effective than traditional physical health teaching in terms of the efficiency of physical health teaching and the degree of physical health knowledge acquisition, respectively. In summary, machine learning-based physical health teaching can substantially improve the efficiency of physical health teaching, enable students to learn more physical health knowledge, and effectively reduce the frequency of students' sports injuries. However, the predictive analysis ability of BP neural network and other techniques cannot reach zero error, the machine learning-based physical health teaching relies on ultra-highly accurate predictive analysis techniques, and improving the predictive analysis ability of machine learning techniques will be the direction of future research.

## Figures and Tables

**Figure 1:** Machine learning-based model for teaching physical health.

**Figure 2:** Neuron structure diagram.

**Figure 3:** BP neural network structure diagram.

**Figure 4:** Classification model diagram of support vector machine.

**Figure 5:** Diagram of the plain Bayesian classification model.

**Figure 6:** Diagram of the Bayesian classification model with expanded tree shape.

**Figure 7:** Graph of students' sports injuries.

**Figure 8:** Graph of students' level of interest in physical education and health learning.

**Figure 9:** Comparison chart of the efficiency of two types of physical health teaching.

**Figure 10:** Graph of students' acquisition of physical health knowledge.

**Table 1:** Table of indicators for evaluating the quality of physical education and health teaching.

Impact indicator	High school	Sophomore	Senior year
Student sports injuries	81%	78%	78%
Students' interest in physical fitness learning	83%	82%	82%
The efficiency of physical health teaching	84%	82%	84%
The acquisition of sports health knowledge	76%	64%	72%
Students' passion for sports	62%	54%	66%
Correcting the odds of a student's athletic misconduct	56%	42%	58%
Average	73.7%	67%	73.3%

**Table 2:** The degree of correlation between evaluation indicators and physical health teaching.

Number of sample groups	Impact indicator	Relevance
1	Student sports injuries	0.264
2	Students' interest in physical fitness learning	0.222
3	The efficiency of physical health teaching	0.233
4	The acquisition of sports health knowledge	0.221
5	Students' passion for sports	0.026
6	Correcting the odds of a student's athletic misconduct	0.034

**Table 3:** Table of results of sample validity analysis.

Evaluation indicators	Physical health teaching based on machine learning	Traditional physical education
Student sports injuries	82.4%	72.8%
Students' interest in physical fitness learning	72.6%	86.2%
The efficiency of physical health teaching	86.2%	83.2%
The acquisition of sports health knowledge	88.4%	78.2%
Average	82.4%	80.0%

**Table 4:** Comparison of the average data of the two approaches to teaching physical health.

Compare items	Physical health teaching based on machine learning	Traditional physical education
Student sports injuries	24.4%	32.1%
Students' interest in physical fitness learning	53.3%	40.3%
The efficiency of physical health teaching	65.2%	49.1%
The acquisition of sports health knowledge	73.2%	63.9%

## Data Availability

The data that support the findings of this study are available from the corresponding author upon reasonable request.

## References

[1] Hodges M., Kulinna P. H., Lee C., Kwon J. Y. (2017). Professional development and teacher perceptions of experiences teaching health-related fitness knowledge. *Journal of Teaching in Physical Education*.

[2] Dunleavy P. T., Sposetti D. M. (2017). Interprofessional peer teaching: physical therapy students teaching dental students to transfer patients. Collaborative healthcare: Interprofessional practice. *Education and Evaluation (JCIPE)*.

[3] Thompson S., Bartram R., Sweeney T., Dias R., Nicholls T. (2020). Bitesized teaching: educational futures for mental health training. *British Journal of Mental Health Nursing*.

[4] Chun C., Yin W. Z. (2017). Mathematical statistics-based university students' physical health conditions and teaching strategies study. *Eurasia Journal of Mathematics Science & Technology Education*.

[5] Bartram R., Dias R., Thompson S. (2017). Bitesized teaching: delivering knowledge of physical health issues in mental health settings. *British Journal of Mental Health Nursing*.

[6] Li F., Wang C., Yue X. (2022). Impact of doctoral student training process fit on doctoral students’ mental health. *International Journal of Mental Health Promotion*.

[7] Song H., Brandt-Pearce M. (2012). A 2-D discrete-time model of physical impairments in wavelength-division multiplexing systems. *Journal of Lightwave Technology*.

[8] Li H. (2020). Analysis of computer teaching pattern based on outlier data mining and machine learning. *Journal of Intelligent and Fuzzy Systems*.

[9] Zhang Y. (2021). Interactive intelligent teaching and automatic composition scoring system based on linear regression machine learning algorithm. *Journal of Intelligent and Fuzzy Systems*.

[10] Hou Y. (2020). Students' emotional analysis on ideological and political teaching classes based on artificial intelligence and data mining. *Journal of Intelligent and Fuzzy Systems*.

[11] Zhang Z., Min H. (2020). Analysis on the construction of personalized physical education teaching system based on a cloud computing platform. *Wireless Communications and Mobile Computing*.

[12] Yang D. M. (2017). Research on college students' individual physical health promotion - based on the perspective of physical education reform. *Agro Food Industry Hi Tech*.

[13] Rubin E., Beuk F. (2021). Emotions and spillover effects of social networks affective well being. *Journal of Organizational and End User Computing (JOEUC)*.

[14] Peijian J., Shimei S., Ning H. (2017). Study of GA-BP neural network method on predicting regional risk of rock burst. *Disaster Advances*.

[15] Jiang Y., Choo K.-K. R., Ko H. (2021). A special section on deep & advanced machine learning approaches for human behavior analysis. *Journal of Information Processing Systems*.

[16] Liu H., Liu J., Wan Y., Xia Y., Guo Z. (2021). Identification of grouting compactness in bridge bellows based on the BP neural network. *Structure*.

[17] Zhang Q., Guo Y., Song Z. Y. (2021). Dynamic curve fitting and BP neural network with feature extraction for Mobile specific emitter identification. *IEEE Access*.

[18] Luo H. (2018). a lithology identification method for continental shale oil reservoir based on BP neural network. *Journal of Geophysics and Engineering*.

[19] Ding H., Jiang X., Li K., Guo H., Li W. (2020). Intelligent classification method for tunnel lining cracks based on PFC-BP neural network. *Mathematical Problems in Engineering*.

[20] Yu H., Gao L., Liao W., Bing Z., Philips W. (2017). An unsupervised convolutional feature fusion network for deep representation of remote sensing images. *IEEE Geoscience and Remote Sensing Letters*.

[21] Yang Y., Demmel J., Czechowski K., Le S., Vuduc R. (2017). Design and implementation of a communication-optimal classifier for distributed kernel support vector machines. *IEEE Transactions on Parallel & Distributed Systems*.

[22] Feng X., Li S., Chao Y., Peng Z., Yang S. (2018). Prediction of slope stability using naive Bayes classifier. *KSCE Journal of Civil Engineering*.

[23] Shirakawa M., Nakayama K., Hara T., Nishio S. (2015). Wikipedia-based semantic similarity measurements for Noisy short texts using extended naive Bayes. *IEEE Transactions on Emerging Topics in Computing*.

[24] Bahr M. W., Edwin M., Long K. A. (2022). Exploratory factor analysis, reliability, and validity of the interventionist knowledge and skills survey. *Psychology in the Schools*.

[25] Kyriazos T. A., Stalikas A. (2019). Alabama Parenting Questionnaire-Short Form (APQ-9): evidencing construct validity with factor analysis, CFA MTMM and measurement invariance in a Greek sample. *Psychology*.

[26] Boudreaux M. J., South S. C., Oltmanns T. F. (2019). Symptom-level analysis of DSM-IV/DSM-5 personality pathology in later life: hierarchical structure and predictive validity across self- and informant ratings. *Journal of Abnormal Psychology*.

[27] Harris G. L. H., Poole G. B., Harris W. E. (2014). Globular clusters and supermassive black holes in galaxies: further analysis and a larger sample. *Monthly Notices of the Royal Astronomical Society*.

[28] Buczak A., Guven E. (2016). A survey of data mining and machine learning methods for cyber security intrusion detection. *IEEE Communications Surveys & Tutorials*.

